# Effects of Gyroscope on Arm Swing and Gait in Healthy Volunteers

**DOI:** 10.1155/2023/6630913

**Published:** 2023-03-15

**Authors:** Meriç Selim Şipal, Elif Yalçın, Aynur Ayşe Karaduman

**Affiliations:** ^1^Physical Therapy and Rehabilitation Hospital, Ankara City Hospital, Ankara, Turkey; ^2^Departmant of Physical Therapy and Rehabilitation, Lokman Hekim University, Ankara, Turkey

## Abstract

**Background:**

Arm swing has a crucial role in gait. It is essential in terms of regulating gait parameters and balance during walking. In the case of bradykinesia, the arms act as a generator to maintain lower extremity movement while walking. The way gyroscopes work makes them useful in arm swings. In this study, the arm swing is facilitated by a new type of gyroscope. As a main purpose, a gyroscope was used to increase arm swing during pendulum exercise and walking.

**Methods:**

Thirty healthy volunteers were included in the study. The study covered three situations. The first evaluation was performed without the gyroscope. The second evaluation was performed while the gyroscope was installed but not activated. The final evaluation was made while the gyroscope was installed and powered up. The effect of the gyroscope on the arm swing was evaluated by the Dartfish®, and the gait was evaluated with the Zebris® force distribution measurement analysis system.

**Results:**

According to the results, the gyroscope increases the arm swing in the pendulum exercise (*p* < 0.05). Furthermore, using the gyroscope, the step width decreased, and the gait cycle time increased (*p* < 0.05).

**Conclusions:**

The gyroscope is suitable for facilitating arm swings in healthy volunteers. This study is essential to demonstrate the effect of a gyroscope on extremity movements for the first time. In the future, a medical device that has the features of a gyroscope can be designed for its use in the treatment of Parkinson's disease and Senile Bradykinesia.

## 1. Introduction

Arm swing has a crucial role in gait. It is essential in terms of regulating gait parameters and balance during walking [1, 2]. This key role gives researchers a means to affect movement patterns. In normal motion, the arms act as a stabilizer to neutralize the dispersed movement [3]. In the case of bradykinesia, arms also act as a generator to maintain movement of the lower extremities while walking [4]. This shows the importance of using the arms as a lever to control human dynamics.

The way the arm swing moves makes gyroscopes very suitable to use as an arm swing facilitator, as gyroscopes can move with minimal contact and restriction.

Gyroscopes consist of a rotating center and a base that move in harmony with the angular velocity of rotation. There are many gyroscope types classified according to principles of physics on which they are based and the technology they contain [5]. In the first half of the nineteenth century, French physicist Jean B. L. Foucault contributed to understanding the orbital movements of the Earth with his experiments, using a pendulum and a gyroscope [6].

For a long time, attempts have been made to convert the circular motion of gyroscopes into planar motion. These trials are generally called the gyroscopic inertial thruster (GIT). Due to the basic qualities of the gyroscopes, studies have been only partially successful [7].

The most rational use of the GIT is not to move the target object directly with gyroscopic force but to change the trajectory of the object by making a critical intervention in the motion pattern. Similarly, the effort to achieve a greater result with a limited effect has been the subject of life in many ways. In sports such as Judo, a small impact on the key point serves as a critical intervention and provides the desired result. This is an excellent example of using the moment of inertia in critical response.

It is known that the slightest change causes an effect on all body segments along the bottom-up kinetic chain. Even a problem such as functional hallux limitus, which affects only the big toe, affects gait kinetics from the bottom up [8]. It is a good example that body kinesiology should be considered as a whole. In this sense, the fact that small interventions can have big results for the body should not be ignored.

Evidence shows that adding weight to the body changes gait parameters and improves postural balance [4, 9, 10]. Also, adding weight to the arms can change arm movements and supports the relationship between extremities during walking [4, 9].

In addition to biomechanical connections, neural connections regulate upper and lower extremity movements. Studies suggest a flexible task-oriented neural coupling between lower and upper extremity muscles [11]. This neural mechanism is called the spinal pattern generator. This reflex pathway, which uses bilateral oscillators to regulate rhythmic movement, is thought to exhibit a residual function in quadripedal locomotion [11, 12]. Since this path is active during walking, it can be said that it is possible to feed the path and change walking parameters by regulating arm swing and vice versa.

The main purpose of this study is to regulate arm swing and gait with gyroscopic motion. This study is important in demonstrating the effect of a GIR on extremity movements. Furthermore, it is preliminary research for a medical device with possible use in Parkinson's disease (PD) and Senile Bradykinesia treatment.

## 2. Methods

The GIT effect was revealed by a new instrument with conventional gyroscopic features. This new gyroscope is named gyroscopic movement facilitator (GMF).

The GMF has an energy source and a minimotor. The rotor speed of the gyroscope can be >2,000 rpm (revolutions per minute) when operated. It maintains speed against internal friction. It uses internal friction as part of the system. Friction contributes to the functional integration of the system.

The total weight of the GMF is 550 g. The length of the wrist connection rope is adjusted as required so that the gyroscope does not touch any part of the body during its use. The stability of the gyroscope also prevents movements outside the required pattern.

The arm swing should be revealed comfortably and naturally while using the GMF. This is possible by using the feedback mechanisms of the GMF as a cue for the movement pattern. The location of the internal friction serves as a pivot of the gyroscopic movement, and the characteristic sound produced by the friction in every oscillation contributes to auditory feedback. Additionally, the GMF has a slight vibration produced by the axial tilt of the gyroscope. This vibration is used as tactile feedback to feed the mental image of the arm swing motion. All feedback mechanisms used in the study are essential for creating an arm swing loop while using a gyroscope.

The upper extremities move in a flexion–extension cycle with rotation as an arm swing [13]. It causes an elliptical orbit. When using the GMF with the arm swing, in every oscillation, the gyroscope keeps its direction looking outward of the elliptical orbit. The gyroscope reveals precessional thrust movement at both ends of the elliptical orbit to maintain the movement pattern. It can be called a “correction reaction,” and it is a result of gyroscopic inertia. Gyroscopic inertia also prevents chaotic motion by preventing irregular motions. Most importantly, the sudden movement created by the acceleration and correction reaction constitutes a thrust at the vertex of the elliptical orbit, and the GMF uses this thrust effect by adding it to the arm swing.

If the gyroscope rotated in a circular orbit instead of an elliptical swing of the arm, the GIT effect would not occur in this way. In the circular orbit condition, the mechanism would rotate constantly on the outer side of the circular orbit due to gyroscopic inertia (Figure 1).

Thirty healthy volunteers over 18 years were included in this study. No inclusion criteria other than age were determined. Those with any joint disease or neurological disease were excluded from the study. This information was questioned in the general evaluation.

Arm swing evaluations were performed in a bent position. Participants were asked to swing their arms with body motion, back and forth like a pendulum, for 1 min (not swing their arms intentionally). This is the definition of a “pendulum exercise” (Codman exercise) [14]. A warm-up walk was performed prior to evaluation. All measurements were repeated twice.

Second, the participants walked on the evaluation track. During walking, participants were asked to focus on walking in general and not try to swing their arms more or less. The walk was made on a track consisting of 11 m, 3 m on the walking analysis platform and 4 m before and after the platform to exclude the acceleration and deceleration phases of the gait. The assessment was repeated twice. In addition, a warm-up walk was performed before the evaluation. A minute of rest is provided between the assessments (Figure 2).

The study covers three situations. The first evaluation was performed without the gyroscope. The second evaluation was performed while the gyroscope was installed but not activated. The final evaluation was made while the gyroscope was installed and powered up. Distinctive marking was used for different trials; the plus sign is given when the mechanism works and the minus sign is given when it does not work (dummy condition for the weight effect). The neutral condition represents the evaluation performed without the gyroscope. Due to the effect of sequential flexion and extension on each other, data were treated as “arm swing,” denoting the sum of flexion and extension.

There is an important detail in the use of the GMF. When the gyroscope is introduced to the user, it is said to be comfortable, as if you were carrying something insignificant or accepting the gyroscope as an extension of your arm. Otherwise, users can suppress gyroscopic features by pacifying their arm movements.

The kinematic analysis of the arm swing was evaluated and recorded using the 2D video analysis method (version 4.2.2, Dartfish, Switzerland). The time–distance characteristics of gait were evaluated with Zebris® force distribution measurement (Medical GmbH, Germany). The Zebris® gait analysis system is a walking path with special sensors that assess the time–distance characteristics of gait [15]. During walking, pressure sensors measure the gait parameters and record them via a computer connection.

All participants have given their informed written consent to participate in the research. This study was approved by the local research ethics board (ethics board approval number: E2-21-135).

Repeated measurement analysis of variance and Friedman analysis were used for the analysis. In the measurements that differ, Bonferroni analysis, or multiple comparison tests, was applied to determine the source of the difference. Data were analyzed using the Statistical Package for the Social Sciences version 23.0 (IBM Corp., Armonk, NY, USA).

Post-hoc power analysis of arm swing measurements in the pendulum exercise revealed that the study power was 99% (G^*∗*^Power, version 3.1.9.4, Universität, Düsseldorf, Germany).

## 3. Results

The mean age of volunteers was calculated as 30.60 ± 6.51. The oldest was 47 years old, while the youngest was 22 years old.

Considering the small number of samples and examining the normality of the values, the Shapiro–Wilk statistic, which gives more reliable results in smaller samples, was used. Looking at the Shapiro–Wilk statistics, it can be seen that the values with *p* > 0.05 show normality, so parametric tests were used. Otherwise, nonparametric tests were used for analysis.

As a result of the repeated measures analysis of variance, significant differences were found between pendulum arm swing measurements. The Bonferroni analysis was applied to determine the source of the difference; it was observed that the mean of the pendulum arm swing (+) measurement was significantly higher than the other measurements. Comparison of arm swing kinematics is summarized in Table 1.

As a result of the Friedman analysis, significant differences were found between walking arm swing measurements. As a result of the multiple comparison analysis applied to determine the source of the difference, it was observed that the mean of the walking arm swing (−) measurement was significantly lower than the other measurements (Figure 3).

As a result of the repeated measures analysis of variance, no significant differences were found between the use of the GMF and other conditions in terms of stride length (*p* > 0.05). In addition, there is a statistically significant decrease in cadence with the use of the GMF compared to other conditions (*p* < 0.05).

As a result of the repeated measures analysis of variance, significant differences were found between step widths in walking measurements. As a result of the Bonferroni analysis applied to determine the source of the difference, it was observed that the means of the step width (+) measurement was significantly lower than the other measurements (Table 2).

As a result of the Friedman analysis, significant differences were found between gait cycle times. As a result of the multiple comparison analysis applied to determine the source of the difference, the gait cycle time (+) was significantly higher than the gait cycle time (neutral) measurement (Table 3).

## 4. Discussion

In the literature, it has been suggested that the arms show mass-damping features and are used to reset the angular acceleration of the whole body [16]. This can be explained by the fact that its center of mass remains higher than the center of mass and acts as a naturally tuned mass damper. So, the arm swing is part of the normal gait pattern to reset the body momentum.

Some studies show that adding extra weight can decrease arm swing [1, 2]. To explain the relationship between adding weight to the arm and decreasing movement, it is necessary to examine the issue in detail. The center of mass of the upper extremity is just above the elbow [17]. Adding any weight proximal to the midpoint would mean shortening the effective length of the arm as a pendulum and increasing the damping of the motion. In that case, the frequency of motion increases, and the swing movement gets dampened. In the study by Pontzer et al. [2], the weight attached proximally to the elbow and the damping of movement that occurred should be considered in this way. It is possible to call this situation a kind of mass-damping effect.

This situation can be compared to using mass-damping pendulums to balance tall buildings. Similarly to adding weight to the proximally attached elbow, a heavy pendulum is positioned to hang from the top floor of the building. During an earthquake, this pendulum dampens the movement of the building by swinging naturally in the opposite direction [18].

In the study by Pontzer et al. [2], 1.8 kg was added to the upper elbow level; and in the study by Donker et al. [1], 1.2 kg was added to the tip of the extremity. The amount of weight used in these studies (1.2–1.8 kg) may have limited the natural appearance of the arm swing motion. The total weight ratio of the arm to the body is 0.049 [19]. Adding 2 kg equates to placing ∼60% of a 70 kg person's arm weight. However, this rate is 15% when 0.5 kg is added to the extremity. Excess weight stretches the supporting structures of the shoulder and may cause increased friction during pendulum movement. As a result, studies showing that the arms swing decreases with the added weight have methodological problems related to the place where the weight is added and the amount of its use.

In contrast, if a suitable weight, for example, 500 g, were attached to the tip of the extremity, it would increase movement, as in the study by Yoon et al. [4]. In this study, since the weight is added to the end of the extremity and the movement is not locked with the excess weight, the mass damping effect did not occur. With the use of the GMF, weight was added to the tip of the extremity to increase its effective length without causing a mass-damping effect.

The contribution of the GMF to arm swing appeared to increase movement during pendulum exercise. The GMF contributes to the arm swing even more than the dummy condition that the gyroscope does not work. The pendulum exercise is a good indicator, as it represents the swing of the arm without being influenced by other body mechanics. The effect that occurs during the pendulum exercise best represents the effect of the GMF.

In the study by Yoon et al. [4], it was shown that arm swing anteversion and retroversion increased with 500 g of arm weight while walking, and this increase continued significantly from the first trial to the last trial. In this study, the use of the gyroscope did not produce significant differences in arm swing during walking but did show greater arm swing compared to the dummy condition. This shows that the functioning of the gyroscope regulates movement and prevents chaotic movement caused by a hanging object.

Arm swing has often been counted as counteracting movement against the swing of the legs in walking [2, 3, 20]. The angular momentum of the lower and upper bodies has been suggested to be equal in opposite directions and the net angular momentum of the body is close to zero [16]. Biomechanically, it is clear that the upper extremities are in a close relationship with the lower extremities. In this way, it can be predicted that if the upper body movements are increased, the lower body movements will be more involved in the movement to reset it.

With the use of the GMF, the gait cycle time increased compared to the neutral condition. Also, stride length did not change with the use of the gyroscope, but the cadence was significantly reduced. The reduction in cadence was revealed using only the gyroscope and not in the dummy condition. It can be said that walking slower without decreasing the stride length is a specific gait pattern that occurs only while using the gyroscope.

The step width with the GMF was significantly lower than the other conditions. Step width and gait cycle time are directly relevant to the gait balance. The reduction in step width and the increase in gait cycle time can be interpreted as an improvement in walking balance. However, if both parameters were decreased, it would be more effective in terms of maintaining balance without decreasing gait speed. As a result, it can be said that a slower and more balanced gait can be achieved with the use of the gyroscope.

It should not be forgotten that the level of the wrist is distal to the center of gravity of the body. In other words, adding weight to the wrist shifts the center of gravity of the body downward. So, adding weight to the distal part of the body means increasing the body's stability. If the ground is taken as a reference, the body can be counted as a reverse pendulum. Thus, as a principle of pendular motion, it can be said that while adding weight to the wrist increases the movement of the small pendulum in the body (arm swing), it reduces the movement of the large pendulum (increases body balance). In other words, the GMF regulates arm swing and gait stability by increasing movement in the small pendulum and decreasing movement in the large pendulum.

Feedback is a useful way to affect body kinematics. The literature shows that verbal instructions or deliberately increasing arm swing help to improve gait parameters in PD [21, 22]. Based on this fact, the effect of the GMF on arm swing was not designed solely through the gyroscopic effect. In addition to the GIT effect, feedback mechanisms played an essential role in this study. Tactile, auditory, and visual feedbacks constitute the feedback system of the GMF. Tactile and auditory feedbacks come from the internal friction and vibration of the gyroscope.

The GMF uses the internal friction of the gyroscope to maintain the gyroscopic multiaxial movement pattern, which also contributes to the integration of the system. At the same time, internal friction serves as part of the feedback mechanism by producing a unique sound during each swing motion. This sound cue is used to ensure the continuity of the movement pattern.

The literature suggests that adding weight to the arm can create sensory input and altered perception that can activate the motor cortex for locomotion [4]. In this study, the weight of the GMF and the vibration created by the gyroscopic structure were used as tactile feedback to increase awareness of movement.

Another type of feedback used in this study is visual feedback. Using gyroscopic thrust movement as visual input simplifies maintaining the closed-loop pattern of the arm swing. Once the integrity of this movement is perceived and adopted, it only remains to repeat and automate the learned motion.

Although there are feedback mechanisms that make it easy to use the GMF, it takes time to get used to it. In the pendulum exercise, the same movement pattern is repeated over and over for a minute. Therefore, the user could better understand what to do and how to use the gyroscope. However, during the gait assessment, the user walked a distance of 11 m only twice. As a result, the user has a limited time to get used to the gyroscope while walking. This is one of the most important reasons why the arm swing was not better with the use of the gyroscope than the neutral condition in walking.

Moderate signs of PD, such as decreased arm swing, stiffness, tremor, and changes in gait pattern, are found in 40% of the elderly population [23, 24]. Thus, it can be said that the potential use of the GMF does not only cover people who already have arm swing disorders. It seems possible to use it in people whose arm swing is slightly reduced and are likely to experience similar problems in the future due to their age. Furthermore, since reduced arm swing is an early symptom of PD, the GMF could facilitate early intervention for movement problems [25].

It is known that a decrease in body dynamics has negative consequences on daily life, such as increased immobility, restriction of community ambulation, and dependence on others [26, 27]. It can be expected that facilitating walking will lead to an increase in daily walking. Furthermore, increasing walking would also improve cardiopulmonary endurance as a secondary effect [28]. In the future, this should be the most important clinical goal for the use of facilitation methods with the gyroscope. In addition, the GMF can be an alternative to using weights in pendulum exercises for frozen shoulder and similar joint problems. Separate, long-term studies are needed for all these subjects.

Although conventional exercise therapy is known to be partially successful in the treatment of neurological diseases, the suggestion of innovative approaches is very important in terms of providing diversity in treatment and strengthening the clinician's hand [29].

As a limitation, the study is based on short-term effects. Long-term effects should be studied. Furthermore, due to the importance of arm swing asymmetry in PD, the gyroscopic effect should be investigated bilaterally in future studies.

## 5. Conclusion

In conclusion, it seems possible to use a medical gyroscopic device based on the characteristics of the GMF in people whose arm swing is reduced. The use of a gyroscope as a movement facilitator has the potential to provide early intervention for hypokinesia that occurs with PD and aging.

## Figures and Tables

**Figure 1:** (a) Pendulum exercise position, (b) difference between the circular orbit and the pendulum orbit, and the acceleration of the gyroscope (elliptical orbit, representing the arm swing with the working gyroscope).

**Figure 2:** Applications of arm swing and gait analysis measurements.

**Figure 3:** Box plots of the distribution of walking arm swing measurements.

**Table 1:** Examination of the differences between arm swing measurements.

Assessments^*∗∗*^	*n*	Mean ± SD	*p*	Difference
Pendulum arm swing (neutral)	30	25.17 ± 10.96	0.000^*∗*^	(+) different from others
Pendulum arm swing (−)	30	23.98 ± 9.15		
Pendulum arm swing (+)	30	32.60 ± 9.99		

SD, standard deviation; (neutral), without gyroscope; (−), gyroscope does not work; (+), gyroscope works;  ^*∗*^*p* < 0.05;  ^*∗∗*^All measurements are in degrees.

**Table 2:** Examination of the differences between step width measurements.

Assessments^*∗∗*^	*n*	Mean ± SD	*p*	Difference
Step width (neutral)	30	12.83 ± 2.49	0.000^*∗*^	(+) different from others
Step width (−)	30	12.37 ± 2.44		
Step width (+)	30	11.67 ± 2.40		

SD, standard deviation; (neutral), without gyroscope; (−), gyroscope is not working; (+), gyroscope is working;  ^*∗*^*p* < 0.05;  ^*∗∗*^All measurements are in centimeters.

**Table 3:** Examination of differences between gait cycle time measurements.

Assessments^*∗∗*^	*n*	Median	Min.–max.	*p*	Difference
Gait cycle time (neutral)	30	1.12	1.02–1.37	0.000^*∗*^	(+) different from (neutral)
Gait cycle time (−)	30	1.13	0.12–1.31		
Gait cycle time (+)	30	1.19	1.09–1.38		

Min., minimum; max., maximum; (neutral), without gyroscope; (−), gyroscope not working; (+), gyroscope working;  ^*∗*^*p* < 0.05;  ^*∗∗*^All measurements are in seconds.

## Data Availability

The data used to support the findings of this study are available from the corresponding author upon request.
